RETRACTED

# PSMB5 Alleviates Ulcerative Colitis by Inhibiting ROS-Dependent NLRP3 Inflammasome-Mediated Pyroptosis

**DOI:** 10.1155/2022/2329904

**Published:** 2022-08-26

**Authors:** Liang Han, Yanping Hao, Xudong Wu, Duanmin Hu

**Affiliations:** ^1^Department of Gastroenterology, Second Affiliated Hospital of Soochow University, Suzhou City, Jiangsu Province, China; ^2^Department of Gastroenterology, Yancheng First People's Hospital, Yancheng City, Jiangsu Province, China

## Abstract

Ulcerative colitis (UC) is a chronic inflammatory disease. Intestinal mucosal injury is a significant factor in UC. Pyroptosis is a kind of programmed cell death induced by inflammatory caspases. Proteasome 20S subunit beta 5 (PSMB5) promotes cell viability. The purpose of this study was to determine the impact of PSMB5 on intestinal mucosal injury and to elucidate the underlying processes in dextran sulfate sodium- (DSS-) induced UC mice. Kunming (KM) mice received 3% DSS for 5 days to induce UC. We collected clinical symptoms, body weight, colon length, and histological changes. MDA (malondialdehyde) and SOD (superoxide dismutase) levels were determined using an ELISA assay. RT-PCR was used to assess the expression of IL-1*β* and IL-18. PSMB5 demonstrated a significant effect against UC by increasing body weight and colon length and decreasing DAI (disease activity index), colon macroscopic damage index (CMDI), histological injury scores, and reactive oxygen species (ROS), MDA, and SOD levels, thereby alleviating histopathological changes and inhibiting oxidative stress. HIEC-6 cells were exposed to lipopolysaccharide (LPS) condition with or without PSMB5, along with caspase-1 inhibitor (Z-VAD-FMK), NLRP3 inhibitor (MCC950), and ROS scavenger N-acetylcysteine (NAC). The viability of the cells, the release of lactate dehydrogenase (LDH), and intracellular ROS generation were determined using assay kits. Western blot analysis was used to determine the levels of NLRP3, ASC, cleaved caspase-1 (p20), pro-IL-1*β*, IL-1*β*, pro-IL-18, and IL-18. PSMB5 overexpression enhanced the inflammatory damage in LPS-treated HIEC-6 cells by activating the NLRP3 inflammasome and mediating pyroptosis, as demonstrated by increased LDH release and lower cell viability, as well as increased expression of NLRP3, ASC, cleaved caspase-1 (p20), IL-1, and IL-18. Meanwhile, NAC protected HIEC-6 cells from LPS-induced damage by reversing the activation of the NLRP3 inflammasome-mediated pyroptosis. In conclusion, PSMB5 may lower HIEC-6 cell susceptibility to LPS and ameliorate UC-induced HIEC-6 cell damage by decreasing ROS generation and hence inhibiting NLRP3-mediated pyroptosis.

## 1. Introduction

Inflammatory bowel disease (IBD) is a chronic inflammatory digestive ailment that comprises Crohn's disease (CD) and ulcerative colitis (UC) [1]. The incidence of IBD is increasing year after year, and it is the most common digestive disorder in the world. Chronic diarrhea, abdominal pain, fever, and weight loss are some of the clinical signs of IBD [2]. If the condition progresses, it can lead to intestinal obstruction, intestinal perforation, and even colon cancer lesions in some cases. It is believed that the lesions of UC originate in the rectum and progress to the proximal colon, causing inflammation of the colonic mucosa and submucosa, as well as other organs [3]. The disease has a high occurrence rate and is difficult to treat or eliminate. The current consensus is that UC is the product of a number of contributing factors.

RETRACTED

Pyroptosis is a sort of planned cell death that has only recently been discovered [4]. The activation of caspase-1 is triggered by inflammasomes, including NLRP3, NLRC4, Nlrp1b, and AIM2, which cleaves pro-caspase-1 into activated caspase-1, promoting the maturation of IL-1*β* and IL-18 precursors into mature interleukin (IL)-1*β* and IL-18, and then mediating pyroptosis, which is important in the development and maintenance of inflammatory responses [5]. This receptor, which resembles a nod, may recognize various stimuli such as PAMPs and DAMPs and activate pro-caspase-1, which then cleaves to form active caspase-1, which ultimately leads to the maturation and production of IL-1*β* and IL-18 [6]. Exogenous stimuli such as LPS and endogenous injury signals such as uric acid and ATP have been shown to activate common pathways, such as reactive oxygen species (ROS) production, that lead to the activation of the NLRP3 inflammasome and the subsequent induction of caspase-1-dependent pyroptosis, according to research [7]. ROS are well-known to have a significant role in the pathophysiology of a variety of inflammatory illnesses, including arthritis [8]. Oxidative stress and mitochondrial dysfunction may both increase the production of ROS, which could accelerate tissue damage and cause it to spread. The production of NLRP3 in response to the priming signal provided by LPS is inhibited by a ROS inhibitor, showing that ROS plays a significant role in the control of NLRP3 gene expression [9]. The excessive accumulation of ROS in the intestinal mucosa of UC patients can be observed, and it has been shown to significantly increase inflammation and tissue damage in these patients [10]. In patients with UC, the levels of IL-1*β* and IL-18 are dramatically elevated. As a result, it is reasonable to assume that UC-induced inflammatory damage is involved in pyroptosis.

RETRACTED

PSMB5 is a protein that is found in the active center of the 20S proteasome and has a total amino acid sequence of 264 amino acids. It exhibits chymotrypsin-like activity, which is one of the three key enzymatic activities of the proteasome system, along with chymotrypsin and trypsin [11]. It performs a proteolytic function by controlling the quantity of particular proteins in the body and eliminating misfolded proteins from the bloodstream [12]. The overexpression of PSMB5 in human lens epithelial cells has been shown to improve the ability of the cells to tolerate oxidative stress and to increase cell viability, according to research [13]. The expression of PSMB5 was considerably reduced in L02 cells that had been damaged by oxidative stress, whereas Nrf2 activation can boost PSMB5 expression [14]. Additionally, PSMB5 has the ability to protect pluripotent human bone marrow stromal cells from oxidative damage [15]. As a result, PSMB5 is a critical target in the fight against oxidative stress.

The activation of the ROS-induced NLRP3 inflammasome, which triggers caspase-1-dependent pyroptosis, is critical in the development of cell damage in diabetic rats [16]. It is uncertain whether the NLRP3 inflammasome, which is triggered by ROS, is also implicated in UC-mediated inflammatory damage. It is also unclear what the relationship is between PSMB5 and NLRP3 inflammasome-mediated caspase-1-dependent pyroptosis in the UC. Using this study, we hope to learn more about the role of PSMB5 in the regulation of NLRP3 inflammasome-mediated caspase-1-dependent pyroptosis in the UC, as well as about the underlying mechanism that causes this inflammatory damage.

## 2. Materials and Methods

### 2.1. Animals and Experimental Design

Male Kunming (KM) mice weighing 20 ± 2 g were supplied by the Experimental Animal Center of Dalian Medical University, Dalian, China. All experimental protocols were authorized by the Animal Care and Use Committee of Second Affiliated Hospital of Soochow University. The mice were housed under standardized circumstances at a temperature of 22–24°C, and 20% humidity with a 12 h light/dark cycle, and they had unrestricted access to standard feeding and water ad libitum. After acclimation for one week, 20 mice were randomly assigned into four groups (*n* =5). Group 1 got regular drinking water alone, while the other three groups (Groups 2-4) received 3% DSS (MW 36,000 to 50,000 kDa, MP Biomedicals LLC, Santa Ana, CA, USA) diluted in drinking water for 7 days to induce UC. Mice in Group 4 were injected 1 *μ*g of PSMB5 plasmid into the tail vein. All mice were killed after 14 days. The length of the colons was measured and then washed instantaneously applying ice-cold physiological saline. One portion of colon tissue was immediately split and fixed in 10% formalin for pathological inspection, while the other sections were preserved at −80°C for Western blotting or RT-PCR analysis.

RETRACTED

### 2.2. Evaluation of Disease Activity Index

Based on body weight, gross rectal bleeding, and stool consistency, the mice were tested daily to assess UC degree. A disease activity index (DAI) score was computed according to a published approach to quantify the disease severity. DAI = (Weight Loss Rate Score + Stool Trait Score + Occult Blood Score)/3.

### 2.3. Colon Histopathology

The length of the colon was measured. Then, a 0.5 cm colon segment was fixed in 10% formalin for 24 h, paraffin-embedded, sliced into 5 *μ*m slices, and stained with hematoxylin-eosin (H&E) for histological investigation. Each sample was evaluated at 40×, 100×, and 400× magnification. Histological scores were provided on a scale as mentioned before.

### 2.4. IHC Staining

Primary antibodies against PSMB5 (Abcam, Cambridge, UK) were used for IHC staining, which were incubated at 4°C overnight before being incubated for 50 min at room temperature with HRP-labeled Goat Anti-Rabbit IgG (H+L) (Servicebio). The antigen-antibody response was visualized using diaminobenzidine (DAB). Microscopy was used to photograph the slides (Olympus BX53). Image Pro Plus 6.0 was used to calculate integrated optical density (IOD) in three or five randomly chosen locations for each group (Media Cybernetics, Inc.).

### 2.5. The Measurement of ROS Production in the Colon Tissue

According to Servicebio's established procedures, dihydroethidium (DHE) was used to identify reactive oxygen species (ROS) in tumor tissue. Fresh frozen colon tissues were embedded in an optimum cutting temperature compound (OCT, Sakura) and sectioned at a thickness of 5 *μ*m thick. After washing, the sections were incubated with DHE dye (Servicebio) for 30 min at 37°C, followed by DAPI for 10 min. A fluorescent microscope was used to view the slides. Image Pro Plus was used to determine the mean fluorescence intensity (MFI) of DHE in three randomly chosen locations for each group.

### 2.6. ELISA

MDA (malondialdehyde) and SOD (superoxide dismutase) levels in colon tissue supernatants were determined using ELISA kits (ProteinTech, China) in accordance with the manufacturer's instructions.

### 2.7. Cell Culture and Transfection

Normal human intestinal epithelial cells (HIEC-6, ATCC® CRL-3266) were cultured in RPMI-1640 media with 10% fetal bovine serum (Gibco, CA, USA) (16000-044, Gibco, CA, USA). Cells were plated into the six-well plate and incubated at 37°C in a humidified atmosphere containing 5% CO_2_. When the density reached around 70%, cells were transfected with plasmids by using Lipofectamine™ 2000 according to the manufacturer's instructions (Thermo Fisher Scientific, MA, USA). After 48 hours, RNA was extracted, and protein was isolated 72 hours post-transfection. The siRNA targeting PSMB5 (5′- TAGCGCGTAGATCTCAGGT-3′, GenePharma, Shanghai, China) or pcDNA3.1-PSMB5 overexpressing plasmids were transfected into cells using LipofectamineTM 2000. Following 48 hours of transfection, cells were harvested.

RETRACTED

### 2.8. Cell Treatment

LPS (L2630, Sigma) was dissolved in deionized sterile water and utilized at a final concentration of 1 *μ*g/ml [17, 18]. Z-VAD-FMK (Sigma, USA), a caspase-1 inhibitor, was dissolved in dimethyl sulfoxide (DMSO) and utilized at a concentration of 50 *μ*M. MCC950 (Selleck, USA) was employed at a concentration of 5 M as an inflammasome inhibitor, and N-acetylcysteine (NAC, Sigma, USA) was utilized at a concentration of 10 mM dissolved in sterile deionized water as a ROS inhibitor.

### 2.9. Cell Viability Assay

CCK-8 was used to assess the vitality of the cells (Dojindo Molecular Technologies, Kumamoto-ken, Japan). After incubation, the cells were gently washed with PBS, and then 10 *μ*L of CCK-8 and 100 *μ*L of fresh medium were added to the cells and incubated at 37°C for another 1 hour. After incubation, the optical density (OD) at 450 nm was determined. The relative cell viability was determined by normalizing the control group's OD450 value.

### 2.10. Detection of Intracellular ROS Level

The production of peroxides was determined using the ROS assay kit (Beyotime, Haimen, China). Stable cell lines (20,000 cells/well) cultivated on collagen-coated glass coverslips were treated for 20 min at 37°C with 10 *μ*M 2,7-dichlorodihydrofluorescein diacetate (DCFH-DA). Following that, the cells were photographed using a laser scanning confocal microscope (Nikon, Japan) at 488 and 525 nm for excitation and emission, respectively. The fluorescence intensity was used as a proxy for ROS production.

### 2.11. LDH Activity Assay

LDH activity in the supernatants was quantified for the purpose of evaluating cell damage using a commercially available LDH assay kit (Jiancheng, Nanjing, China) in accordance with the manufacturer's instructions, as previously described.

### 2.12. Western Blotting

Total proteins were isolated from colonic tissues and cells using a standard extraction reagent including the protease inhibitor (KANGCHEN; Shanghai, China). Protein concentrations were determined using the BCA kit (Beyotime, China), as directed by the manufacturer. Equal quantities of proteins (30 *μ*g) were separated by SDS-PAGE gel and then transferred to a PVDF (Millipore, USA) membrane. The membranes were blocked for 1 hour at room temperature with 5% skim milk in PBS, followed by 24 hours at 4°C incubation with primary antibodies against anti-PSMB5, anti-cleaved caspase-1 (p20), anti-pro-IL-1*β*, anti-IL-1*β*, anti-pro-IL-18, anti-IL-18, anti-NLRP3, anti-ASC, and GAPDH. Following that, the blots were washed three times with TBST (10 min for each wash) and incubated for 1 hour with anti-rabbit IgG (1 : 10,000). Finally, immunoreactive bands were visualized and quantified using an Odyssey infrared scanning system (LI-COR Biosciences, USA).

RETRACTED

### 2.13. Real-Time RT-PCR

GAPDH was used as a housekeeping gene. The sequences of specific primers are as follows. GAPDH-F: CCTTCCGTGTCCCCACT, GAPDH-R: GCCTGCTTCACCACCTTC; RIP3-F: TCCAGGGAGGTCAAGGC; RIP3-R: ACAAGGAGCCGTTCTCCA.

The experimental protocols followed those previously described. Trizol was used to extract total RNA (Invitrogen, CA, USA). Hifair II 1st Strand cDNA Synthesis SuperMix was used to synthesize cDNA (Yeasen, Shanghai, China), then configure the Real-Time PCR reaction device and execute the qPCR software according to the instructions included with Hieff UNICON® qPCR SYBR Green Master Mix (Yeasen, Shanghai, China): step 1- 95°C, 30 sec; step 2- 95°C, 5 sec; step 3- 60°C, 20 sec; step 4- 72°C, 20 sec; repeat steps 1-3 repeat 40 cycles. As a housekeeping gene, GAPDH was employed. The sequences of specific primers are as follows: GAPDH-F: CCTTCCGTGTCCCCACT, GAPDH-R: GCCTGCTTCACCACCTTC; RIP3-F: TCCAGGGAGGTCAAGGC, RIP3-R: ACAAGGAGCCGTTCTCCA; PSMB5-F: CATTGTTGCAGCGGATTCCC, PSMB5-R: TAGATTCGACACTGCCGAGC. The gene expression in each group was analyzed using 2^−*ΔΔ*CT^ method.

### 2.14. Statistical Analysis

All analyses were performed using the SPSS 23.0 software package (SPSS Company, Chicago, IL, USA). Data were presented as means ± standard deviation (SD). Differences between the two groups were evaluated using a two-way analysis of variance (ANOVA) followed by Bonferroni's post hoc test. Nonparametric data and continuous variables were analyzed using the Kruskal–Wallis test and one-way ANOVA, respectively. The two-sided *P* values less than 0.05 were deemed significant statistically.

## 3. Results

### 3.1. PSMB5 Improves Body Weight, DAI, and Colon Length for DSS-Induced UC Mice

The mice were treated with 3% DSS for 5 days to induce UC. When compared to control mice, both the DSS-alone treatment group and the DSS-joint vector treatment group exhibited a substantially elevated DAI score (Figures 1(a) and 1(b)). Compared to the DSS group, the DSS-joint PSMB5 vector group had a higher DAI score. The DSS-alone treatment group and the DSS-joint vector group had a considerably lower weight change than the control group, notably in the first seven days, when their weight change was negative (Figure 1(b)). After 3 days, the weight growth resumed a favorable trend. On the ninth day, the weight change of mice in the DSS-joint PSMB5 vector group was negative, but rebounded to a positive level after one day. Additionally, the weight change of mice in the DSS-joint PSMB5 vector group was greater than that in the DSS-alone treatment group and the DSS-joint vector group on day 12 compared to the DSS-alone treatment group and the DSS-joint vector group. Colon length was significantly shorter in DSS-treated mice than in control mice. PSMB5 overexpression ameliorated DSS-induced colon length shortening (Figure 1(d)). DSS enhanced CMDI in mice treated with DSS, but overexpression of PSMB5 decreased CMDI in DSS-treated animals (Figure 1(d)).

RETRACTED

### 3.2. PSMB5 Mitigated Colon Tissue Injury in DSS-Induced UC Mice

In the control group, intact colonic epithelial cells and crypt structure, as well as full goblet cells, were detected. All DSS-treated mice had severe lesions, including loss of colonic epithelial cells, crypt structural deformation, and extensive inflammatory cell infiltration. However, as compared to all DSS-treated mice, the colons of UC mice transfected with PSMB5 plasmids revealed less structural damage, less inflammatory cell infiltration, and only minimal crypt deformation (Figure 2(a)). Additionally, transfection of PSMB5 resulted in a substantial decrease in DSS-induced histological damage scores (Figure 2(b)). Following that, IHC staining revealed that DSS dramatically decreased PSMB5 expression in colon tissues, while transfection of PSMB5 overexpression boosted PSMB5 expression in colon tissues of DSS-treated animals (Figure 2(c)). Taken together, our findings indicated that PSMB5 effectively preserved colon tissue and decreased the morphological alterations in colon tissue caused by DSS.

### 3.3. PSMB5 Could Counteract the Oxidative Stress and Inflammatory Cytokine Secretion Induced by DSS

DSS may raise the amount of ROS, increase the amount of MDA, and decrease the amount of superoxide dismutase (SOD) to produce oxidative stress (Figures 3(a)–3(c)). Meanwhile, DSS-treated mice showed significantly higher levels of IL-1*β* and IL-18 than the control group (Figures 3(d) and 3(e)). However, oxidative stress and inflammatory cytokine release were significantly reduced in the DSS-joint PSMB5 overexpression group than in the DSS-treated group.

### 3.4. PSMB5 Reduced Pyroptosis Mediated by NLRP3 Inflammasome in DSS-Treated Mice

We next evaluated the amounts of cleaved caspase-1 (p20), pro-IL-1*β*, IL-1*β*, pro-IL-18, IL-18, NLRP3, and ASC in colon tissues to see whether they were involved in NLRP3 inflammasome-mediated pyroptosis in DSS-treated mice. PSMB5 expression was significantly greater in the DSS-joint PSMB5 overexpression group than in the other DSS groups (Figures 4(a) and 4(b)). As shown by the results, DSS may activate the NLRP3 inflammasome by raising the levels of NLRP3, ASC, and capase-1 in comparison to control groups (Figures 4(c)–4(e)). DSS treatment resulted in increased production of pro-IL-1*β*, IL-1*β*, pro-IL-18, and IL-18 (Figures 4(f)–4(i)). Following that, we discovered that overexpression of PSMB5 inhibited pyroptosis induced by NLRP3 inflammasome activation in response to DSS stimulation.

RETRACTED

### 3.5. LPS-Medicated Decreased PSMB5 Was Associated with NLRP3 Inflammasome Activation and ROS

To begin, HIEC-6 cells were transfected with siRNA targeting PSMB5 to reduce PSMB5 expression (Figures 5(a) and 5(b)). Then, we discovered that LPS greatly raised the level of NLRP3, but the caspase-1 inhibitor (Z-VAD-FMK) decreased it (Figure 5(c)). Additionally, siRNA-PSMB5 overexpression enhanced NLRP3 expression by more than twofold in cells treated with LPS. The multiprotein complex composed of NLRP3, ASC, and caspase-1 is the NLRP3 inflammasome, which is the primary mechanism of pyroptosis and inflammation after cell damage. The particular molecular mechanisms by which Z-VAD-FMK and MCC950 decrease LPS-induced pyroptosis and influence PSMB5 expression were further investigated. As shown in Figure 5(d), Z-VAD-FMK and MCC950 reduced NLRP3 inflammasome activation in LPS cells by downregulating caspase-1, NLRP3, and ASC protein levels. The two inhibitors also dramatically reduced mature IL-18 and IL-1*β* protein expression. These findings indicate that Z-VAD-FMK and MCC950 may protect cells from LPS-induced damage by suppressing NLRP3 inflammasome activation, lowering oxidative stress, preventing activated caspase-1-induced pyroptosis and inflammation, and increasing PSMB5 expression.

### 3.6. PSMB5 Inhibited the ROS-Dependent NLRP3 Inflammasome to Protect against LPS-Aggravated Pyroptosis

PSMB5 knockdown exacerbated the cell-inhibiting, LDH-increasing, and ROS-enhancing effects of LPS, while NAC restored these effects (Figures 6(a)–6(d)). As shown in Figure 6(e), PSMB5 silencing elevated LPS-activated NLRP3 inflammasome activation and mature IL-18 and IL-1*β* levels, while NAC reversed PSMB5 silencing's heightened effects on NLRP3 inflammasome activation and IL-18 and IL-1*β* secretions.

## 4. Discussion

Pyroptosis is a factor in the development of inflammatory illnesses such as IBD [19]. Inflammatory caspases are markedly increased in IBD. Cholecalciterol Cholesterol Emulsion can cure IBD by reducing pyroptosis [20]; mesalazine and corticosteroids also reduce pyroptosis of intestinal epithelial cells [21]. As a result, more research into the function and mechanism of pyroptosis in UC is required. We created a UC mouse model with 3 percent DSS and discovered that DSS-treated mice showed severe colon tissue injury, elevated inflammatory cytokines, and activated oxidative stress and the NLRP3 inflammasome. To summarize, DSS-induced UC triggered an inflammatory caspase-medicated NLRP3 inflammasome, whereas DSS-stimulated ROS buildup can also activate the NLRP3 inflammasome to drive inflammatory cascades. Activated NLRP3 inflammasomes activate caspase-1, resulting in the production of mature IL-1*β* and IL-18 and, as a result, pyroptosis. DSS produced pyroptosis, which exacerbated colon tissue injury, according to the findings.

RETRACTED

PSMB5 controls cell proliferation and protects bone marrow mesenchymal stem cells (BMSCs) from oxidative stress injury, allowing them to remain cytoactive and limit cell aging [22]. In this study, we discovered that animals in the DSS-joint PSMB5 overexpression group had less colon tissue injury and weight change than mice in the DSS-treated group as a whole. PSMB5 overexpression reduced DSS-induced oxidative stress and NLRP3 inflammasome activation. It demonstrated that PSMB5 could prevent the advancement of UC.

We employed lipopolysaccharide- (LPS-) treated cells to replicate UC-medicated cell damage to examine the mechanism of PSMB5 in UC-mediated pyroptosis. The main conclusion of our investigation was that LPS at a concentration of 1 g/ml increased cell damage by activating the NLRP3 inflammasome and pyroptosis via the ROS/NLRP3-mediated caspase-1 pathway. PSMB5 inhibition exacerbated LPS-induced cell damage. Z-VAD-FMK inhibits casapase-1, and NAC inhibits ROS. Z-VAD-FMK and NAC treatment may alleviate LPS-induced PSMB5 expression inhibition and protect cells from LPS-induced damage by reducing the NLRP3 inflammasome and pyroptosis, which was probably connected with lower ROS production. To the best of our knowledge, this is the first study to look into the mechanism of PSMB5 in pyroptosis, which was linked to ROS-dependent NLRP3 inflammasome-activated caspase-1 to cause pyroptosis.

ROS functions as a second messenger to activate inflammasomes and has been identified as a key mechanism for NLRP3 inflammasome activation [23]. It is a frequent NLRP3/caspase-1 complex activator that is involved in pyroptosis. To maintain a balance of ROS formation and clearance, antioxidant enzymes can remove ROS during cell metabolism under normal conditions. When ROS accumulates indefinitely and the endogenic antioxygen defense mechanism is unable to clear it in time, it causes oxidative stress, cellular diseases such as increased lipid peroxidation, and cell death [24]. UC increased oxidative stress and caused an increase in cytokine production in the intestine [25]. Furthermore, ROS triggers inflammatory pathways [26]. In the current work, we discovered that NLRP3 inflammasome activation increased considerably in a ROS-dependent manner to promote pyroptotic cell death in cells stimulated with LPS. We also discovered that NAC suppressed ROS generation, which reduced the activation of the NLRP3 inflammasome and thereby alleviated LPS-induced cell damage. ROS was found to be an activator of the NLRP3 inflammasome and caspase-1-dependent pyroptosis in LPS-treated cells [27]. Furthermore, inhibiting ROS is an effective therapy for LPS-induced cell damage. PSMB5 knockdown may prevent NAC's protective effects on LPS-treated cells. It demonstrated that PSMB5 was a NAC action target for inhibiting pyroptosis.

RETRACTED

Finally, our findings revealed that DSS and LPS exacerbated cell damage by targeting the ROS/NLRP3 inflammasome pathway and the downstream activated caspase-1 and IL-1*β* pathway to promote pyroptosis and inflammatory responses. Our findings further indicated that PSMB5 can reduce pyroptosis in H9C2 cells by suppressing ROS/NLRP3 inflammasome activation, suggesting that it may be a new therapeutic target for reducing cell harm during UC.

## Figures and Tables

**Figure 1:** PSMB5 improves body weight, DAI, and colon length for DSS-induced UC mice. (a) The disease activity index (DAI). (b) The body weight change. (c) Colon length. (d) The colon macroscopic damage index (CMDI). All data are expressed as mean ± SD (*n* =5). ^∗^*p* < 0.05.

**Figure 2:** PSMB5 mitigated colon tissue injury in DSS-induced UC mice. (a) Histopathology (magnification 40x, 100x, 400x). (b) Histopathological scores. (c) IHC analysis of PSMB5 (magnification 40x, 100x, 400x). All data are expressed as mean ± SD (*n* =5). ^∗^*p* < 0.05, experiment group compared to the control group.

**Figure 3:** PSMB5 could fight DSS-induced oxidative stress and inflammatory cytokine secretion. (a) Dihydroethidium (DHE) analysis of ROS level. (b and c) ELISA analysis of MDA and SOD levels. (d and e) RT-PCR analysis of IL-1*β* and IL-18 levels. All data are expressed as mean ± SD (*n* =5). ^∗^*p* < 0.05.

**Figure 4:** PSMB5 reduced pyroptosis mediated by NLRP3 inflammasome in DSS-treated mice. (a) Images from Western blotting. (b) Western blot analysis of PSMB5, cleaved caspase-1 p20, pro-IL-1*β*, IL-1*β*, pro-IL-18, IL-18, NLRP3, and ASC at protein level. All data are expressed as mean ± SD (*n* =5). ^∗^*p* < 0.05.

RETRACTED

**Figure 5:** LPS-medicated decreased PSMB5 was related to the activation of NLRP3 inflammasome and ROS. PSMB5 expression at protein level (a) and mRNA level (b) was detected by Western blot and RT-PCR assay in siRNA targeting PSMB5 transfected HIEC-6 cells. (c) Western blotting for PSMB5 expression under LPS and Z-VAD-FMK conditions. (d) Western blot analysis of PSMB5, cleaved caspase-1 p20, pro-IL-1*β*, IL-1*β*, pro-IL-18, IL-18, NLRP3, and ASC expressions under LPS and Z-VAD-FMK conditions or LPS and MCC950 conditions. All data are expressed as mean ± SD (*n* =5). ^∗^*p* < 0.05 and ^#^*p* < 0.05.

**Figure 6:** PSMB5 protects against LPS-aggravated pyroptosis by inhibiting ROS-dependent NLRP3 inflammasome under LPS and NAC conditions, in siRNA-PSMB5 transfected HIEC-6 cells, (a) CCK8 analysis of cell viabiltiy, (b) LDH activity assays of the LDH release, (c and d) DCFH-DA assay of the ROS production, and (e) Western blot analysis of cleaved caspase-1 p20, pro-IL-1*β*, IL-1*β*, pro-IL-18, IL-18, NLRP3, and ASC expressions. All data are expressed as mean ± SD (*n* =5). ^∗^*p* < 0.05 and ^#^*p* < 0.05.

## Data Availability

The data of this study is available upon reasonable requests from the corresponding author.
